This article has been retracted.

# Emotion Analysis Based on Neural Network under the Big Data Environment

**DOI:** 10.1155/2022/7123079

**Published:** 2022-09-27

**Authors:** Jing Zhou, Quanju Liu

**Affiliations:** Department of Computer School, Huanggang Normal University, Huanggang, Hubei 438000, China

## Abstract

Aiming at the problems of poor emotional tendency prediction effect and low utilization of syntactic information, this study proposes a big data sentiment analysis method based on neural network. First, the BERT model is used to vectorize the input data to reduce the semantic loss when the data is vectorized; then the word vector is input into the bidirectional LSTM encoder to obtain data features. Finally, the representation of the attention layer is used as the final feature vector for sentiment classification, reducing the influence of irrelevant data. The experimental results show that the method has high accuracy, recall, and F1 value and can effectively improve the accuracy of fine-grained sentiment classification of ambiguous texts.

## 1. Introduction

Text sentiment analysis is an interdisciplinary problem in the fields of information retrieval, natural language processing, and artificial intelligence, which can clarify the emotional content of text description [1]. Most of the previous sentiment analysis is sentence implementation analysis of chapter structure and paragraph structure, but with the increasingly significant needs of users, the roughness of sentiment analysis at this level is obvious. A paragraph or a sentence only expresses an emotional attitude, which cannot accurately describe the content that users want to know. Sentiment orientation analysis is the core work of text sentiment analysis, which is to judge the sentiment orientation of texts containing subjective information. According to the number of affective categories, the affective tendency analysis task could be divided into dichotomous-category (positive/positive, negative/negative), tripartite-category (positive, negative, neutral), and multicategory (happy, excited, sad, angry, etc.) tasks. Since fine-grained target/aspect sentiment analysis needs to accurately analyze all aspects of sentiment orientation mentioned in the text and can provide more comprehensive and detailed sentiment information, which is also the paper's research hotspot and future trend of text sentiment orientation analysis.

There are researchers to research on text classification of emotional problems. Fukushima et al. [2] proposed based on fine-grained multichannel convolution neural network text sentiment analysis method; this method can dig deep semantic information in text and text sentiment analysis, but this method is not applicable to text sample more. Liu et al. [3] proposed a multilanguage text emotion analysis method integrating attention mechanism. The advantage of this method lies in the realization of multilanguage text emotion analysis, but the classification accuracy of ambiguous text emotion needs to be optimized. The analysis methods based on machine learning and emotion dictionary mainly label the text features manually and then construct machine learning classifier to obtain the final emotion trend of the text. Liu et al. [3] constructed an adaptive emotion dictionary by combining corpus and dictionary to enhance the judgment ability of text emotion polarity. Lin et al. [4] used the combination of support vector machine and text frequency in Chinese reviews to determine the emotional trend of review texts. Although the above methods have achieved good results, the performance of sentiment analysis is highly dependent on the text features manually annotated, and the applicability of the method is far lower than that of the neural network-based method. In general, the existing methods are difficult to extract text features with sentiment discrimination, and the accuracy of sentiment analysis is not high. Therefore, it is necessary to study a more efficient sentiment analysis model, which can achieve efficient feature extraction and higher precision sentiment analysis.

In natural language processing, unstructured text content needs to be transformed into a vectorized form, so that the computer can recognize and calculate, and the vectorized data can be reused. To solve the task of natural language processing, text should be structured and digitized and expressed as word vector, which is convenient for computer processing. Early word vector representation based on word bag model is high dimensional and sparse, and its feature expression ability is weak, which is not conducive to feature extraction [5]. The proposed distributed representation based on word embedding makes it possible for deep learning to be used in short text sentiment analysis. Word embedding technology maps text into low-dimensional real vectors by learning a large amount of corpus [6]. The word vector is then input into the deep neural network to automatically extract context features, and the final text representation is used for sentiment orientation analysis [7]. Word embedding technology is still developing and some pretrained language models are proposed to measure the similarity between words. Word2Vec was proposed in 2013 [8], GloVe in 2014 [9], OpenAIGPT in 2016 [10], ELMo (embeddings from language models) [11, 12] and BERT (bidirectional encoder representation from transformers) were proposed in 2018 [13, 14], and Transformer-XL [5] and XLNet [13] based on Transformers [15] architecture were proposed in 2019. The pretraining models commonly used in short-text affective orientation analysis include Word2Vec, GloVe, and BERT.

To sum up, most machine learning models will cause information loss when processing emotional texts when the average vector of above context or aspect words or the first (CLS) vector after splicing is used as the subfeature [16]. In addition, in the scenario of implicit aspect words, the method based on aspect words embedding and fusion of position-weighted information is no longer applicable. Therefore, this paper studies a BERT representation based attention network that uses LSTM model to fuse syntactic information [17]. The model as input, the text sentence through structure (CLS) is used more than token embed mode to reduce the processing long text information loss, at the same time by combining attention mechanism memory deep aspects of network structure to capture the sentence semantic representation, to enhance the model in the implicit aspects under the term and the long text sentiment analysis in terms of performance [18]. In order to improve the accuracy of text sentiment analysis, a bidirectional gated loop network was used to train text features with shared weights, and the text features were combined with context information. The graph attention network was used to process the text features with syntactic information, which made full use of syntactic information and strengthened the interaction between different nodes in the text [19].

The structure of this paper is as follows: chapter 2 introduces neural networks, fine-grained analysis, and other related theories; chapter 3 introduces the construction of sentiment text analysis model in detail; chapter 4 is the experimental part of this paper, which is used to verify the effectiveness of the model; in the conclusion part, the research content and innovation of this paper are summarized in detail and the future work is prospected.

## 2. Related Work

### 2.1. Neural Network

Traditional machine models need to transform text into bag of words before analysis, then into TF-IDF matrix, and then classification, while using neural network model can make text extract features and classification by itself and can obtain better ability than traditional machine learning model.

Convolutional neural network was proposed after Fukushima, a famous Japanese neural network expert, established a new generation of neural cognitive machine model based on the concept of receptive field. The main characteristic of CNN is that the neural network can accurately capture locally related targets and has been widely used in actual image processing. In mathematics, it is generally called (*f*∗*g*)(*n*), the convolution of *f* and *g*. *f* and *g* are integrable functions. In the continuous case, the convolution is defined as:

(1) $$\begin{array}{c} \left(f*g\right)\left(n\right)=\int_{‐\infty }^{\infty }f\left(t\right)g\left(n-t\right)dt, \end{array}$$

where *f* and *g* are integrable functions. Convolution in the discrete case is defined as:

(2) $$\begin{array}{c} \left(f*g\right)\left(n\right)=\int_{\text{t}=‐\infty }^{\infty }f\left(t\right)g\left(n-t\right). \end{array}$$

At the physical level, the system's output at a particular moment is determined by the previous common output. Kim in 2014 for the first time put forward the text—the convolutional neural network (CNN) applied in classification of emotional work, including shard of vocabulary is in the Text into after preprocessing, after word vector tools into the word vector as the convolution of the neural network input, the model of training need to add text data to the emotional category labels. The results obtained after model training can be compared with the samples before processing, so as to achieve the effect of text classification.

In the CNN structure, the input layer sends the text into the hidden layer in the form of a two-dimensional matrix, but the comment text is one-dimensional data, so the CNN convolution uses one-dimensional convolution. This model needs to use the convolution kernel to hide the input data and deliver it to the calculation matrix when inputting the word vector for each layer. The size of the convolution kernel and the word vector should be relative when calculating in the matrix. The extraction formula for the convolution layer is as follows.

(3) $$\begin{array}{c} C_{i}=f\left(w*x+b\right), \end{array}$$

where *f* is the activation function, *w* is the weight matrix, and *b* is the bias vector. After the convolution operation, there is the pooling layer. The function of the pooling layer is mainly to denoise the words that participate in the training and filter out the elements that do not need to participate in the training. The essential purpose of pooling operation according to the characteristics of the convolution layer has been extracted, the range has a more detailed secondary features which are extracted, output in pooling operation is usually the result of the maximum or average in the local area after the extraction operation of strong characteristics of the original vocabulary was preserved, but it can also cut off the useless information, The purpose of this is to make the network more stable and has stronger anti-interference ability.

Finally, a fully connected Softmax layer outputs the binary polarity of the comment text. Convolutional neural network has many outstanding features, such as strong local perception ability, sharing of extracted parameters, information collection of multikernel convolution, and semantic extraction of various lengths, which is said to be indispensable in text classification.

The main function of the recurrent neural network RNN model is to process the data with sequence, and it has great advantages in the processing of nonlinear sequence such as text. Its characteristic is that the output of the current moment includes the output of the previous moment, and the model of the previous moment can carry out continuous memory of the information by means of cyclic preservation. This function can be said to provide “memory” for RNN. The structure of RNN neural unit is shown in Figure 1.

If there are *n* words in the input data, then the system will logically output *n* neurons. In general, the hidden layer is composed of multiple circulating neural units, so in the calculation of RNN, there will be multiple intermediate data. The following formula can be used to calculate the cyclic neural unit. The current output result and the implicit *ht* can be calculated by input *X*_*t*_ and the implicit state of the last node. The probability output of the calculated result is combined with Softmax function to complete the category prediction.

(4) $$\begin{array}{c} S_{t}=f\left({ux}_{t}+{ws}_{t-1}\right), \end{array}$$

(5) $$\begin{array}{c} h_{t}=g\left(V*S_{t}\right). \end{array}$$

The input data is represented by *X*, *X*_*t*_ represents the word vector received by the cell at time *t*, *S*_*t*_ represents the memory of the sample at time *t*, and the value of *S*_*t*_ not only depends on *X*_*t*_ but also depends on *s*_*t*−1_. *H*_*t*_ is the output of the current cell *t* time; *u* is the weight of input sample, *w* is the weight of memory, *V* is the weight of output sample; *f* and *g* are activation functions, Relu, Sigmoid, and other functions can be activated by *f*, Softmax function can be activated by *g* function. For natural language processing, its essence is carried out in accordance with the time order, so the relationship between the text within the words are arranged according to time order. The model structure can provide a good combination of context, if the time sequences with growth, so the distance information is easy to forget, if you want to deal with the distance information. Then it will take a long time, which is likely to cause gradient explosion and disappearance of problems.

LSTM is a model based on recurrent neural network [20]. The advantage of recurrent neural network model is that it can persistently store feature information. This property makes the model prone to the problem of gradient disappearance if it fails to learn the information with a long feature distance in the back propagation. After in-depth study of the above problems, such as Hochreiter one after the experimental summary introduced a new generation of LSTM model. The basic structure of the new model is based on neural network, but its main characteristic is increased in every unit around the door of the three kinds of structure as shown in Figure 2.

This LSTM network model can be formed after the combination of multiple time-sequence modules. Such three-gate layout exists in each sequential module, and the three gates are input *i*_*t*_, forgetting *f*_*t*_, output *O*_*t*_, and cell state *C*_*t*_, respectively. Tanh is the hyperbolic tangent function, *σ* is sigmoid function, ⊕ is element-level addition, and ⊗ is element-level multiplication. *X*_*t*_ is the input of the current moment and *h*_*t*−1_ is the output of the hidden layer at the previous moment.

The main function of the input gate is to select the information to be added. Its operation principle is to combine the information to be updated with the current time series and finally input the information into the cell state. The formula of the input gate is:

(6) $$\begin{array}{c} i_{t}=\sigma \left(W_{i}*\left[h_{t-1},x_{t}\right]+b_{i}\right), \end{array}$$

(7) $$\begin{array}{c} C_{t}^{\text{'}}=\tanh\left(W_{c}*\left[h_{t-1},x_{t}\right]+b_{c}\right), \end{array}$$

where *W* is the weight and *b* is the deviation. The main function of the input gate is to control the state of the current node. The state control information is based on the input information of the previous moment. If you want to skip the current node for control, you can also directly complete the input and transfer to the next node. The purpose of the forgetting gate is to control how much content of the cell state of the previous layer needs to be forgotten. The formula of the forgetting gate is as follows:

(8) $$\begin{array}{c} f_{t}=\sigma \left(W_{f}*\left[h_{t-1},x_{t}\right]+b_{f}\right), \end{array}$$

(9) $$\begin{array}{c} C_{t}=f_{t}*C_{t-1}+i_{t}\times C_{t}^{\prime }. \end{array}$$

To activate this function, you need to use the Sigmoid function to complete, where the output results are only 0 and 1, 0 means that the output results are completely forgotten, on the contrary, 1 means that the output results are completely remembered. When processing text information, the main function of the forgetting gate is to forget the previous subject and complete the memory of the new subject. When the cell state is updated, the output can be carried out. The cell state *C*_*t*_ will judge the output results in the long- and short-term network, and the formula is as follows:

(10) $$\begin{array}{c} O_{t}=\sigma \left(W_{O}*\left[h_{t-1},x_{t}\right]+b_{O}\right), \end{array}$$

(11) $$\begin{array}{c} h_{t}=O_{t}*\tanh\left(C_{t}\right). \end{array}$$

The main working steps of the output gate are the following points, the first is to calculate the cell state *C*_*t*_, then the output part will be output after the Sigmoid layer calculation, and then the state *C*_*t*_ will pass through the tanh layer. The final output result is obtained by the tanh layer, and the Sigmoid layer output results in the multiplication operation. It can be seen that LSTM plays a good role in solving the trouble of gradient disappearance or explosion in the process of information transmission, which enables the model to master the dependent information of nonlinear sequence in the process of learning.

### 2.2. Fine Size Analysis

Aspect-level sentiment analysis, also known as attribute-level sentiment analysis, which aims to give the emotional polarity of a text from a specific angle. For example, in this task, the scores of scenic spots and hotels are divided into six aspects: overall, service, location, facilities, sanitation, and cost-performance, which makes it difficult for the traditional sentence-level sentiment analysis method to directly complete the task. In recent years, research on fine-grained emotion analysis focuses on deep learning methods. Hu et al. [21] constructed a Recursive Neural Network based on dependency tree. Xu and Qian [12] introduced the Attention Mechanism into LSTM and proposed ATAE-LSTM model, which can make full use of attribute information. Lane et al. [22] proposed TD-LSTM and TC-LSTM models for fine-grained sentiment analysis, which divided sentences into left and right parts according to context. Devlin et al. [23] proposed a deep memory network architecture, which judges the importance of each context word to a specific attribute through the Attention Mechanism, and realizes the interaction between attribute and context by using the attention mechanism. Socher et al. used BERT-LSTM to form sentence-level memory representation, and makes corresponding weights based on the relative positions of each word and attribute, so that the same sentence has different representations under each attribute. In addition, fine-grained sentiment analysis tasks are widely used in multimodal fields to model image-text pair interaction and fusion, and the model effect is more than that of a single text mode [24]. With the BERT model's breakthrough achievement in 11 downstream tasks of natural language processing, the Pretrain/FineTune model architecture has triggered a boom in the research of natural language processing [25]. However, the fine-grained emotion analysis model based on BERT cannot achieve good results on the data set involved in this task, which is embodied in early over-fitting and low accuracy of binary classification.

## 3. Model Building

Bert model can effectively improve the vectorization speed of data and reduce semantic loss. The BERT model does not use the traditional left-to-right or right-to-left language model for pretraining, but innovatively uses the Masked Language model (MLM) and the next sentence prediction task for pretraining [26]. MLM tasks are designed to train deep bidirectional features so that word representations can better integrate with context [27]. The next prediction task is to enable the model to understand the relationships between sentences. In this way, the word vector obtained by BERT not only implies the features between context words but also can capture some sentence-level features. BERT's most important module is the bidirectional transformer code structure. Transformer is a structure proposed by Lappas [28]. For the input text, it conducts model by adopting self-attention mechanism and full connection layer completely rather than uses RNN or CNN for feature extraction [29, 30].

### 3.1. Bidirectional LSTM Coding Layer

The bidirectional LSTM coding layer is composed of two parallel LSTM layers, namely, the forward LSTM layer and the reverse LSTM layer, respectively. BiLSTM layer adds reverse LSTM model on the basis of LSTM model to get forward hidden state and backward hidden state [31, 32]. By splicing forward and backward state vectors, the final output is to make the recognition result more accurate. The forward LSTM combines with the backward LSTM to form BiLSTM. On the basis of the one-way data flow in the LSTM network, the reverse data flow is added, and there is no connection between the forward hidden layer and the backward hidden layer, which effectively solves the problem of LSTM intelligently extracting sequence features in a single direction. Formulas (12)–(17) show the calculation of hidden state *h*_t_.

(12) $$\begin{array}{c} i_{t}=\delta \left(W_{wi}w_{t}+W_{hi}h_{t-1}+W_{ci}c_{t-1}+b_{i}\right), \end{array}$$

(13) $$\begin{array}{c} f_{t}=\delta \left(W_{wf}w_{t}+W_{hf}h_{t-1}+W_{cf}c_{t-1}+b_{f}\right), \end{array}$$

(14) $$\begin{array}{c} z_{t}=\tanh\left(W_{wc}w_{t}+W_{hc}h_{t-1}+b_{c}\right), \end{array}$$

(15) $$\begin{array}{c} c_{t}=+f_{t}c_{t-1}+i_{t}z_{t}, \end{array}$$

(16) $$\begin{array}{c} o_{t}=\delta \left(W_{wo}w_{t}+W_{ho}h_{t-1}+W_{co}c_{t}+b_{o}\right), \end{array}$$

(17) $$\begin{array}{c} h_{t}=o_{t}\tanh\left(c_{t}\right), \end{array}$$

where *i*, f, and *o* are input gate, forgetting gate, and output gate, respectively, *b* is the bias term and *w*_(•)_ is the parameter matrix.

In order to automatically extract entity features, a hidden transformation layer was added to construct a hidden state marker matrix, and the reserved part of information was determined by forgetting gate [33]. The forward LSTM layer is encoded *x*_*t*_ by considering the previous information of *x*_*t*_ from the word segmentation vector *x*_1_ to *x*_*t*_, and the output is denoted as *h*_*t*_. Similarly, the reverse LSTM layer encodes *x*_*t*_ by considering the posttext information of *x*_*t*_ from the word segmentation vector *x*_*n*_ to *x*_*t*_, and the output is denoted as *h*_*t*_ . Finally, Formulas (18) and (19) join *h*_*t*_ and *h*_*t*_ to represent the information of no. *t* participles coding.

(18) $$\begin{array}{c} h_{t}=\left[h_{t}⊕h_{t}\right]\in R^{2de}, \end{array}$$

where ⊕ represents vector connection and *d*_*e*_ is one-way LSTM network dimension. For input *S*, the output of this layer is:

(19) $$\begin{array}{c} h=\left(h_{1},h_{2},\cdots ,h_{n}\right)\in R^{2de\times n}. \end{array}$$

Output *h* in the next layer is the model input. After getting the sequence of context in comprehensive coding, LSTM structure is also used to generate tag sequence, which is called decoding. The decoding layer adopts one one-way LSTM layer, called LSTMd layer, whose structure is shown in Figure 3. While detecting the tags of the word segmentation *x*_*t*_, decode layer's input is: context representation vector *M*_*t*_, which is obtained by participles *x*_*t*_ from bidirectional LSTM coding layer. *T*_*t*−1_ represents the predicted label of previous neurons, *c*_*t*−1_^(2)^ represents the value of previous neurons, *h*_*t*−1_^(2)^ represents the previous hidden vector before decoding layer, and the final output *x*_*t*_ is predicted label vectors *T*_*t*_. Formulas (20)–(26) represent LSTMd decoding layer.

(20) $$\begin{array}{c} i_{t}^{\left(2\right)}=\delta \left(W_{wi}^{\left(2\right)}h_{t}+W_{hi}^{\left(2\right)}h_{t-1}^{\left(2\right)}+W_{ti}T_{t-1}+b_{i}^{\left(2\right)}\right), \end{array}$$

(21) $$\begin{array}{c} f_{t}^{\left(2\right)}=\delta \left(W_{wf}^{\left(2\right)}h_{t}+W_{hf}^{\left(2\right)}h_{t-1}^{\left(2\right)}+W_{tf}T_{t-1}+b_{f}^{\left(2\right)}\right), \end{array}$$

(22) $$\begin{array}{c} z_{t}^{\left(2\right)}=\tanh\left(W_{wc}^{\left(2\right)}h_{t}+W_{hc}^{\left(2\right)}h_{t-1}^{\left(2\right)}+W_{tc}T_{t-1}+b_{c}^{\left(2\right)}\right), \end{array}$$

(23) $$\begin{array}{c} c_{t}^{\left(2\right)}=f_{t}^{\left(2\right)}c_{t-1}^{\left(2\right)}+i_{t}^{\left(2\right)}z_{t}^{\left(2\right)}, \end{array}$$

(24) $$\begin{array}{c} o_{t}^{\left(2\right)}=\delta \left(W_{wo}^{\left(2\right)}h_{t}+W_{ho}^{\left(2\right)}h_{t-1}^{\left(2\right)}+W_{co}^{\left(2\right)}c_{t}^{\left(2\right)}+b_{o}^{\left(2\right)}\right), \end{array}$$

(25) $$\begin{array}{c} h_{t}^{\left(2\right)}=o_{t}^{\left(2\right)}\tanh\left(c_{t}^{\left(2\right)}\right), \end{array}$$

(26) $$\begin{array}{c} T_{t}=W_{ts}h_{t}^{\left(2\right)}+b_{ts}, \end{array}$$

where *i*, *f*, and *o* are input gate, forgetting gate, and output gate, respectively, *b* is the bias term and *w*_(•)_ is the parameter matrix.

For the input *M*, the output of this layer is the vector sequence of prediction labels, the equation is as shown below.

(27) $$\begin{array}{c} T=\left\{T_{1},T_{2},\cdots ,T_{n}\right\}\in R^{d_{d}\times n}, \end{array}$$

where *d*_*d*_ is the LSTMd network dimension.

The 1 × 1 convolution kernel is set to *a*(*y*), *b*(*y*), and *c*(*y*) to complete cross-channel information fusion of text fine-grained emotional features.

(28) $$\begin{array}{c} a\left(y\right)=V_{a}y, \end{array}$$

(29) $$\begin{array}{c} b\left(y\right)=V_{b}y, \end{array}$$

(30) $$\begin{array}{c} c\left(y\right)=V_{c}y, \end{array}$$

where *V*_*a*_, *V*_*b*_, and *V*_*c*_ belong to capsule network parameters; *a*(*y*) and *b*(*y*) can be used to calculate feature similarity of text fine-grained emotion and construct attention mask, and *c*(*y*) can be used to construct the masked model's characteristic image. *Y* belongs to the text fine-grained emotion feature value. The similarity operation method of *r*_*ij*_ and attention mask operation method of *δ*_*ij*_ are as follows:

(31) $$\begin{array}{c} r_{ij}=a\left(y_{i}\right)\left(y_{i}\right), \end{array}$$

(32) $$\begin{array}{c} \delta_{ij}=\frac{\exp\left(r_{ij}\right)}{\sum_{i=1}^{M}\exp\left(r_{ij}\right)}. \end{array}$$

*y*_*i*_ represents the eigenvalue which index in text fine-grained emotional features is *i*. *i* and *j* represent the feature index value; *r*_*ij*_ can calculate the similarity of index *j* position eigenvalue which corresponds to the index *i* position eigenvalue. Normalization will be implemented to *δ*_*ij*_, and calculate the global similarity response value of the eigenvalue of the index *j* position, so as to establish the attention mask matrix. The attention matrix can be obtained through the normalization of the function, and the input end can be associated with the word to be predicted. The output is the weight matrix of each word and the weighted sum of the attention matrix, and the weight is the importance of each input word to the output result.

### 3.2. Text Fine-Grained Emotion Self-Attention Feature Computing

In the case of limited computing power, attention mechanism is the main means to solve the problem of information overload. It is a resource allocation scheme to allocate computing resources to more important tasks. The computing formula of text fine-grained emotional self-attention features is:

(33) $$\begin{array}{c} z_{j}=\overset{M}{\underset{i=1}{\sum }}\delta_{ij}c\left(y\right), \end{array}$$

(34) $$\begin{array}{c} x_{j}=\beta z_{j}+y_{i}, \end{array}$$

where *M* is the number of text fine-grained features, *z*_*j*_ is the self-attention eigenvalue of text fine-grained emotion in position *j* of mask feature index, the weight parameter is *β*, *x*_*j*_ is the self-attention feature of fine-grained emotion of text, index *i* position text fine-grained emotional self-attention eigenvalue is *y*_*i*_.

We use attention mechanism to increase the weight of important information which can better get the intrinsic relevance of semantic information and allocate the weight to get the information of context better. And meanwhile, we use Graph convolutional neural network to extract the feature of triple emotion by the end-to-end which can realize sentiment analysis.

The attention mechanism is used to calculate the correlation coefficient between node *j* and node *i* in the set, and the linear transformation formula is as follows:

(35) $$\begin{array}{c} e_{ij}=\text{LeakyReLU}\left(a\left({Wx}_{i},{Wx}_{j}\right)\right) \end{array}$$

where *a* is the inner product operation of node correlation coefficient.

In order to make the *e*_*ij*_ coefficients easy to compare on all the entities of the set, the coefficients are normalized.

(36) $$\begin{array}{c} a_{ij}=soft\max\left(e_{ij}\right)=\exp\left(e_{ij}\right)/\underset{k\in N_{i}^{r}}{\sum }\exp\left(e_{ik}\right), \end{array}$$

where *a*_*ij*_ is the influence degree of neighborhood node *j* on *i*.

Finally, the normalized weight coefficient *a*_*ij*_ is used to calculate the forward hiding state of node *i*.

(37) $$\begin{array}{c} \overset{⟶}{h_{i}}=relu\left(\underset{j\in N_{i}^{r}}{\sum }\alpha_{ij}{Wh}_{j}\right). \end{array}$$

Similarly, $N_{\overset{⟶}{j}}^{r}$ set uses the same attention mechanism to obtain the backward hidden state $\overset{⟵}{h_{i}}$ of the corresponding node *i*. The eigenvector learning of node *i* comprehensively considers the effects of all its neighborhood nodes on node *i*.

## 4. Experimental Analysis

### 4.1. Experimental Environment Setting

The experimental hardware environment was set as Win10 + Ubuntu1604 dual system, 16 GB memory, GTX1080 graphics card, Intel Core i7 CPU, 1 T hard disk, and Python2.7 programming language and Java toolkit natural language processing tool were used in MATLAB simulation software for comparison experiment. The experimental parameters are set as follows: input dimension seq-length parameter is 128, training set batch-size parameter is 64, test set batch-size parameter is 8, and training learning rate is 2 × 10^−5^. To prevent over-gradient explosions during training, the gradient clamp parameter is set to 5, and the dropout technique is used to prevent over-fitting, with a value of 0.5. To test the proposed method, accuracy (P), Recall (R), and F1 value (F1) were used. The efficiency of the model can be evaluated by integrating the advantages of the four indicators, and the performance of the model can be better evaluated by using the high discrimination ability of the accuracy rate for negative samples, the recognition ability of the recall rate for correct samples and the robustness of the F1 score. The formula is shown below.

(38) $$\begin{array}{c} \text{Accuracy}=\frac{\text{TP}+\text{TN}}{\text{TP}+\text{TN}+\text{FN}+\text{FP}}\times 100\%, \end{array}$$

(39) $$\begin{array}{c} R=\frac{\text{TP}}{\text{TP}+\text{FN}}\times 100\%, \end{array}$$

(40) $$\begin{array}{c} F1=\frac{2\times \text{TP}}{2\times \text{TP}+\text{FP}+\text{FN}}\times 100\%. \end{array}$$

*TP* represents the text in the model as kind of sample that can be correctly predicted as category, *TN* was represented by the negative samples in the text model that can correctly predict negative category, *FP* representative is the negative samples in the text model that can predict wrong category, *FN* representative is the negative samples in text model can predict negative category mistake. The text fine-grained emotion in a chat system is classified, and the text fine-grained emotion types are joy, sadness, surprise, anger, fear, and disgust in turn. Import the chat records in this chat system into MATLAB software, and there are 3000 chat records of six text fine-grained emotions, each emotion text is 500. The dataset used was collected in the form http://kahlan.eps.surrey.ac.uk/savee/Download.html. The detailed settings are shown in Table 1.

The proposed method [2] and literature method [3] were used to conduct text fine-grained emotion classification at the same time. The classification effects of the three methods on the six text fine-grained emotion classification of chat records are shown in Figures 4–6.

It can be seen from Figures 4–6 that the blue bars represent the accuracy, recall, and F1 value of the classification results of the proposed method, which are all greater than 95%, which are 8%-10% higher than that of the method in reference 2, and 10%-13% higher than that of the method in reference 3, showing high accuracy of sentiment analysis. It can be seen that this method is effective for fine-grained sentiment classification of multiple texts.

## 5. Conclusion

Aiming at the problem that the existing text sentiment analysis models fail to make full use of syntactic information and have poor prediction effect of sentiment trend, this paper proposes a big data sentiment analysis research based on neural network. Firstly, the BERT model is used to quantize the word direction of text data. Then feature extraction of word vector is carried out in an end-to-end form to ensure that contextual semantic information is not lost. Finally, fine-grained sentiment analysis of text is realized through attention mechanism. The model constructed in this paper can extract more emotion discriminative features and improve the accuracy of text sentiment analysis.Experimental results show that this model is superior to traditional machine learning and neural network models. In future research, the accuracy of sentiment analysis will be provided from two aspects of constructing sentiment analysis templates and improving network models.

## Figures and Tables

**Figure 1:** Structure diagram of RNN neural unit.

**Figure 2:** LSTM neural network diagram.

**Figure 3:** BERT model diagram.

**Figure 4:** Comparison results of accuracy rate.

**Figure 5:** Comparison results of recall rate.

**Figure 6:** Comparison results of F1 values.

**Table 1:** Experiment text setting.

Emotional types	Number of training texts/unit	Number of test texts/unit
Joy	350	150
Sad	350	150
Surprise	350	150
Anger	350	150
Fear	350	150
Hate	350	150

## Data Availability

The dataset can be accessed upon request.
